This article has been retracted.

# Ecological Landscape Design and Evaluation in Public Charging Facilities for Electric Vehicles

**DOI:** 10.1155/2022/3010851

**Published:** 2022-06-29

**Authors:** Yang Yu

**Affiliations:** Academy of Fine Arts, Weifang University, Weifang, Shandong 261061, China

## Abstract

The deterioration of the environment in the 21st century has made environmental issues one of the most severe tests for modern society. With this comes a change in energy structure from high-carbon to low-carbon direction, and electric vehicles are gradually developing into the darling of a city with low-carbon transportation and safe travel. This paper carries out a systematic analysis of landscape design and environmental protection in the development of new energy electric vehicle charging facilities in urban habitat. By categorizing the content and provisions of published domestic and international standards, new requirements for standardization are obtained, including barrier-free design, electromagnetic radiation, child safety protection, and urban landscape integration. Among them, ecological landscape public charging facilities can enhance the overall quality of urban environment. This paper analyzes the necessity of landscape design in charging facilities, explores the ecological concepts extended by macroscopic landscape design principles and the problems of public charging facilities, and proposes a design and evaluation method of ecologically landscaped public charging facilities based on hierarchical analysis and neural networks. The hierarchical analysis method is introduced to establish a landscape design assessment index system, and then a neural network is introduced to describe the characteristics of electric vehicle charging, and the landscape design assessment learning samples are trained to establish a landscape design assessment model. Finally, a comparison experiment is conducted with other landscape design assessment methods using specific examples, and the results show that the proposed method has more obvious advantages in ecological landscape public charging facility design assessment with high accuracy, faster landscape design assessment, charging efficiency, and environmental protection.

## 1. Introduction

The landscape compatibility problem in public charging facilities foreign studies mainly focuses on the number of charging facilities' fixed capacity and site selection, without considering its function as a building and the building itself into the landscape mechanism and other aspects. As a kind of public service facility with high sustainability and energy ratio, most of the studies on charging facilities focus on functional characteristics, grid mechanism, and operation management, but there is a lack of studies on the characteristic expression of landscape design in charging facilities. Background and trend of landscape reference in public charging facilities: Under the current environmental problems, the use and exploration of sustainable energy has become one of the ways to solve the problems, and charging facilities are expanding under the call of new energy [1–3]. New energy charging facility landscape architecture is a new energy charging facility architecture integrated with aesthetic and artistic design, which can meet people's dual demand for low-energy consumption and architectural aesthetics of the building. In recent years, the development rate of new energy charging facility landscape architecture has been increasing, the design research of new energy charging facility landscape architecture has become a hot spot, and landmark new energy charging facility landscape architecture is emerging. Therefore, it is necessary to review the development background and research history of new energy charging facility landscape architecture, summarize the development of new energy charging facility landscape, and propose the method of new energy charging facility landscape architecture. The existing public charging space has a single set of supporting facilities, grid technology restrictions, and spatial landscape problems, while at this stage the exploration of functionality is much more than the exploration of landscape. In terms of form, the base station extends outside the space in the form of rows of trees with a canopy, providing a resting space and creating a quiet environment. Functionally, while satisfying the demand for fast charging, the space is also designed with landscape references to achieve a harmonious coexistence between man and nature. The superfast charging station superimposes landscape performance based on meeting the needs of functional use, as a type of landscape architecture. From the development trend, the future use of landscape design for charging facilities has become a general trend. The Vinci diagram of the new demand analysis path for standardization of charging facilities in ecological landscapes is shown in Figure 1.

In Figure 1, we analyze the new demand for standardization of charging facilities in ecological landscapes, which mainly includes three aspects: (1) Content of charging facility standards. To meet the latest development trend of electric vehicles, charging facilities need to be designed according to the latest standards. (2) New demands of ecological protection. (3) New demands of landscape design of charging facilities. The popularity of electric vehicles to enhance the ecological protection of society, set point facilities are also an important component of the electric vehicle industry chain and need to further enhance ecological protection. New energy vehicle charging device can be divided into fast and slow charging. Slow charging is the use of AC charging device to input single-phase AC power, the output of the car AC power, but not directly used in the new energy vehicle storage device, and the use of charging devices to achieve the purpose of charging for new energy vehicles. Slow-charging devices can also be combined with the specific use of each type, to be divided into public charging and home charging, where home charging is generally a small-output power, power is usually within 2.8 kW, so the charging time is relatively long, but the cost design is small, so many residents are favored, but the public charging power is relatively high, but the highest power must be within 7.5 kW. The charging time is shorter than that of home charging [4–6]. In addition, in the design and construction of equipment, the construction of JIATO charging equipment is relatively easy and less costly, so it can be well used in construction. Fast charging is a generally used DC mode to charge, which belongs to the battery charging type; there are many manufacturers of this mode charging device; there will be differences between the maximum output power, basically must be suitable to control between 22 kW and 220 kW. In addition, priority should be given to DC equipment of good-quality brand, which can well bear the output voltage and current at the same time, and because of its relatively large variation within the interval, it can generally be used in various models of new energy vehicles so as to achieve the actual needs of various types of new energy vehicle charging, and the installation method of new energy vehicle fast charging device basically adopts the floor type [5].

The existing charging facilities lack reasonable expression of landscape design factors and are not given much attention in this field. The use of urban fragmented space while relying on the urban road network reflects the ecological concept, and the landscape architecture is reasonably planned according to the geographical location, materials, and grid structure. First, for geographical location, the materials of the ultra-fast charging station are collected from its nearby forest park, utilizing the sustainability of the building materials, and the ecological concept is reflected everywhere in the future maintenance of the base station with zero waste and docking of the materials, and the main building materials are considered for future maintenance, while the complexity of the surrounding road network extension from the route also determines its embodiment in functional applications [6]. The location of the base station makes use of the urban debris space, forming a transition space between the city and nature. More importantly, the use of debris space creates a prerequisite space for the harmonious development of man and nature in an urbanized city. Architecture in ecology becomes a carrier of human activities and landscape environment. Second, for the use of materials, the sustainability of wood is constantly reflected in the landscape architecture, fitting the ecological concept and rational planning of sustainability and the fixed capacity of facilities. The main body of local materials highlights the ecological concept of landscape design embodied in the building itself, while the use of materials is also the basis for the charging facilities reflecting the principles of landscape design [7]. The main contributions of this paper include the following: (1) analyzing the existing charging facilities' lack of reasonable expression of landscape design factors, which are not paid attention to in this field. (2) To obtain ideal landscape design and environmental protection effect and evaluation results of electric vehicle public charging facilities, this paper designs hierarchical analysis method and neural network landscape design effect assessment method, which has the advantages of hierarchical analysis method and neural network and overcomes their disadvantages. (3) The results of simulation experiments show that the method in this paper obtains ideal results for the evaluation of the design effect of ecological landscape public charging facilities, and the efficiency of landscape design effect evaluation is also obvious. Moreover, the efficiency of landscape design effect assessment is significantly better than the landscape design effect assessment methods of hierarchical analysis method and neural network.

## 2. Related Work

### 2.1. Ecological Landscape Public Charging Facilities

*Landscape Design Environmental Protection Electric Vehicles*. With the development of clean energy and the promotion of the concept of sustainable development, electric vehicles have gradually become the mainstream transportation. The large number of electric vehicles put into use has reduced environmental pollution and saved energy, but it also brings its charging problem. Charging piles, as an important charging place for electric vehicles, seriously affect the development of electric vehicle industry and the convenience of car owners with their cars [8].

Therefore, it is necessary to plan the site selection, construction capacity, and charging network of charging piles. Power battery performance such as mass specific energy, volume specific energy, charging multiplier, and so on has an important impact on the development of EV charging facilities. Specific energy determines the range of electric vehicles (the driving range of one charge) and charging multiplier determines the charging time. In this paper, we believe that the promotion of electric vehicles can be divided into 3 stages: demonstration, public welfare, and commercial operation. The characteristics of charging facilities planning are different in different stages. In the demonstration stage, the electric vehicle technology is not yet fully mature, and the market mechanism to promote the development of electric vehicles in a sustainable way has not yet been formed. The charging facility planning in the demonstration stage can be regarded as the recent planning. At this stage, EV technology is developing rapidly, but it is still at a low level and there are hidden bottlenecks, such as safety factors; the total number and proportion of EVs at this stage are still relatively low and the economy is not high. The development mode is to rely on government subsidies and lead the propaganda of acceptable charging EVs, which can be expanded to electric buses, public vehicles of large enterprises and institutions, and a few social vehicles. This stage of charging facilities planning can be regarded as medium-term planning. At this stage, the technology of electric vehicles is basically mature, and the total amount of electric vehicles has reached a certain scale and the variety of electric vehicles is relatively rich. At this stage, the economy of electric vehicles is equal to or even surpasses that of fuel vehicles, and the development mode is mainly market driven. The planning of electric vehicle charging facilities at this stage can be regarded as long-term planning.

The basic framework of the habitat standardization system for electric vehicle charging facilities is shown in Figure 2. In this paper, a systematic analysis of the current situation and demand for common standardization of new energy electric vehicle charging facilities in urban habitat is carried out. Firstly, two research methods, content analysis and semistructured questionnaire research, were identified, and the logical analysis path was “induction-deduction” [9–11]. Then, two independent coders categorized the contents and clauses of published domestic and international standards by content analysis, summarized eight types of standardization needs, and compared the missing contents of domestic standards from international standards. Finally, a semistructured questionnaire survey was used to collect the factors that the public thinks need to be included in the consideration of the habitat environment in addition to the existing contents of the standards. The results of the standard code comparison and questionnaire survey show that the current domestic standard system for electric vehicle charging facilities already covers (1) site planning, (2) installation arrangement, (3) environmental requirements, (4) fire safety, (5) energy saving and environmental protection, (6) lighting requirements, (7) noise impact, (8) signs and markings, and other eight aspects of the habitat environment. The four new requirements not yet covered are (9) barrier-free design, (10) electromagnetic radiation, (11) child safety protection, and (12) urban landscape integration. The results of the standard code comparison and questionnaire survey show that the current domestic standard system for electric vehicle charging facilities already covers (1) site planning, (2) installation arrangement, (3) environmental requirements, (4) fire safety, (5) energy saving and environmental protection, (6) lighting requirements, (7) noise impact, (8) signs and markings, and other eight aspects of the habitat environment [12–14].

Public charging facilities at home and abroad account for the background status public charging facilities; that is, public charging stations are a sustainable energy supply facility derived from the current energy structure transformation. New energy vehicles tend to improve the development of energy utilization as the main means, and their charging facilities should be on the same level of hard functionality. In terms of architecture, the open building structure is supposed to be an extension of the space division. Taking the fast-charging station as an example, the basis of functional embodiment extends to the public landscape, and the addition of landscape elements to a certain extent complements the industry, focusing on the symbiosis of architecture and environment and the co-topology of the environmental planning industry chain. Second, the principle of scientific nature of landscape design materials. The choice of materials should also fit the characteristics of sustainable development of charging facilities, the reality of the environment in the material of the facility site has not considered the ecological concept, or even the facility site is under the open air. In terms of materials, the materials age and fall off due to the long-term environment in the open air, which shortens the service life of the materials. Therefore, the choice of materials should consider the influence of external factors, and at the same time, the choice of materials should pay attention to echoing the environment of the facility place. The material selection of the facility space should be combined with the material qualities, environment, and other external objective factors, based on the ecological concept, scientific selection of materials, reasonable protection of landscape architecture, and the principle of scientific should be used to configure landscape materials [15–17]. In the design, the charging station is shown in the form of anthropomorphic trees, and the modular construction method makes the charging station scalable and can perform a “forest” according to the needs. In the use of materials, to reflect the form of the base station, trees selected by the Nature Conservancy were used, and the toughness of the wood meets the requirements to a certain extent, while the attachment of solar panels is ensured [18, 19].

### 2.2. Artificial Intelligence and Landscape Design

With the continuous development and improvement of China's economy, people's living standards are constantly improving, families and public places have carried out some landscape design, landscape design can bring people a more comfortable feeling, and each person has different requirements for landscape design, so the landscape design effect needs to be accurately assessed to better provide people with the best living, working and leisure environment, therefore, landscape design effect assessment has been the focus of people's attention. For landscape design effect assessment, domestic and foreign research institutions have conducted in-depth research, and there are many effective landscape design effect assessment methods. The current landscape design effect assessment method is divided into two kinds of qualitative analysis and quantitative analysis, among which the most representative qualitative analysis method is the hierarchical analysis method, which is based on the landscape design effect assessment indexes; according to the weights of various indicators to the landscape design effect assessment results, the method is relatively simple and belongs to the linear modeling method, while the landscape design effect and evaluation indexes are a nonlinear mapping relationship, resulting in the deviation of landscape design effect assessment is relatively large, and the practical application value is low; the most representative quantitative analysis method is artificial neural network, such as RBF neural network, BP neural network, limit learning machine network, and so on. The artificial neural network has strong nonlinear modeling ability and gets better landscape design effect assessment results. Since landscape design effect assessment is very complex, single hierarchical analysis method and neural network both have their own shortcomings and cannot describe landscape design effect comprehensively and accurately, so landscape design effect assessment faces great challenges [20].

With the concept of developing clean energy and promoting sustainable development, electric vehicles have gradually become the mainstream transportation. Although the large number of electric vehicles put into use has reduced environmental pollution and saved energy, it also brings its charging problem. Charging piles, as an important charging place for electric vehicles, seriously affect the development of electric vehicle industry and the convenience of car owners with their cars. Therefore, it is necessary to plan the site selection, construction capacity, and charging network of charging piles. Landscape scheme design and quality evaluation is divided into subevaluation and overall evaluation where subevaluation is more rational and tends to focus on whether the specific functions of the landscape scheme are reasonable or not, but overall evaluation is also important; it is often a comprehensive evaluation of the landscape scheme by experts based on their own experience. In the past, we often encountered the following situation: every indicator of the landscape scheme is at a medium level, but the total score is low; while some schemes only have a few indicators but score high and other indicators score average, but the total score is high. This fully illustrates that there is a nonlinear relationship between the overall quality of the landscape and the evaluation factors. In this paper, a BP neural network model is used to explain the nonlinear relationship between the quality of natural ecological river landscape schemes and their evaluation factors [20, 21].

Landscape ecological planning is the practical activity of using the principles of landscape ecology to solve ecological problems at the landscape level, which concentrates the application value of landscape ecology, and it is especially significant to apply it to the urban fringe areas with fragile ecology and complex landscape pattern changes. Landscape ecological planning can be understood as follows: based on regional natural, social, and economic information, from a macro, overall, and comprehensive perspective on the regional landscape pattern to make dynamic planning, in order to optimize the structure, protect the ecological balance, and promote the sustainable development of the region. The landscape pattern can be reflected by a set of landscape indices, so the landscape ecological planning process is essentially a nonlinear mapping process, that is, a nonlinear mapping relationship between various topographic factors and various disturbance effects (especially the role of human) and a set of landscape indices. The artificial neural network method that has emerged at home and abroad in recent years can perform large-scale parallel processing of information, is good at association, generalization, analogy, and reasoning, and can extract regular knowledge from a large amount of raw or statistical data, which is very suitable for quantitative research of landscape ecological planning. With the development of artificial neural network technology, researchers have designed a variety of neural network models, which describe and simulate the biological neural system at different levels from different perspectives and are applied in various fields, of which 80%–90% of the artificial neural network models use BP networks or its variant forms, reflecting the best part of artificial neural networks [22, 23].

*The Embodiment of Landscape Design Principles in Facilities*. First, the extension of landscape design in space is tackled. In the existing charging facilities, the landscape of the facility and the building space are separated, and the landscape environment design mostly exists in the external environment [24]. The comfort given by the landscape cannot be extended to the facility body, and the functionality of the space monolith and the landscape environment are out of place. At the same time, in the limited facility space, the planning of landscape design has limitations, and the landscape guided by the principle of natural environment compatibility is extended in the facility. This time, we need to reflect the principle of extension of landscape design, not only in the space inside and outside the environment, but also in the landscape design of plants, visual angle, and landscape carrier extension [25]. In short, the audience's visual angle and sensory experience in the public charging facilities will not have a greater sense of difference when they are extended outside the facilities. Take the high-speed tram charging station as an example; the open space design extends the landscape from internal to external natural space, and the use of pavilion structure extends the tree canopy from the top of the charging station, truly integrating the facility with the landscape, and thus extending the internal environment of the base station to the external environment [26]. Meanwhile, in terms of vegetation, the surrounding plants are mainly local greenery species that can be selected in cooperation with natural resources conservation, and the plant configuration is also an extension from nature to architecture. As mentioned above, the material of the base station is collected from the nearby forest park, which extends from the environment to the facility so that the audience can feel the public charging facility and the environment in the space without any difference. In contrast, the current charging base stations do not consider the extension of landscape design in the space, and the internal and external environments often fail to achieve harmony, and the peripheral environment is only used as green decoration, and the use of the site is more a reflection of function [27].

## 3. Methods

### 3.1. Ecological Landscape Charging Facility Site Selection Model

The overall model structure is shown in Figure 3. To make more reasonable and full use of electric energy resources, optimize charging station area configuration and maximize people's charging demand for electric vehicles, a maximum cut-off model for electric vehicle charging stations is constructed to maximize the service range and charging efficiency of charging stations.

(1) Model assumptions: It is assumed that electric vehicle trips are mainly distributed on the shortest route between the origin and destination. In a transportation network, suppose there are *n* nodes; then there are *n*^*∗*^(*n* − 1) shortest routes. The set of shortest routes between two places is *C*={*C*_1_, *C*_2_,…*C*_*n*^*∗*^(*n* − 1)_}, the length of the shortest route is *Dc*, and *Nc* is the set of nodes on the *c*th shortest route. Assume that the traffic flow on each route can be determined. That is, the traffic route network is deterministic, and the road traffic flow on each route is stable without considering the effect of individual road construction or building. Assume that the traffic route network is a network system, where the set of nodes is *N*={*n*_1_, *n*_2_,…*n*_*n*_}, the set of edges is *A*={*a*_1_, *a*_2_,…*a*_*n*_}, *Q* is the number of charging stations set up, and *R*_*i*_ is the flow of electric vehicles on *a*_*i*_. *H*_max_ is the maximum distance between stations. Define two 0–1 variables, located on the path of *a*_*i*_ to set charging stations; then *x* = 1, otherwise 0; located on the shortest route to plan at least one charging station, *y* = 1, otherwise 0. Assume that there is an upper limit to the number of charging posts in a single charging station. One charging station may not be able to meet the charging demand of all users. Let the charging station have charging piles *f* units, and *f* denotes the number of charging piles installed in charging station *i*.

(2) Modeling:

(1) $$\begin{array}{c} Max\sum_{a_{i}\in A_{c}}R_{i}x_{i}, \end{array}$$

(2) $$\begin{array}{c} \sum_{i-1}^{n}x_{i}=n,\\ D_{c}\times \left(1-y_{c}\right)\leq H_{\max}, \end{array}$$

(3) $$\begin{array}{c} y_{c},x_{j}\in \left\{0,1\right\}. \end{array}$$

The objective function is the maximum traffic flow intercepted; the constraint is the total number of *n* charging facilities installed; the constraint is the maximum capacity of charging facilities not exceeding *S*; the constraint indicates that the user can still charge the electric vehicle during the remaining trips. The constraint indicates that the decision variable takes the value of 0 or 1.

(3) Algorithm solving: Ant colony algorithm refers to an optimization algorithm that simulates the foraging behavior of ants to find the optimal path. By identifying a series of solutions to be optimized as the solution space of feasible solutions, the ant colony algorithm is driven by the pheromone and iterates in a continuous loop to find the optimal path under the influence of positive feedback mechanism and then obtains the optimal solution of the problem. The algorithm is mainly applied to the assignment problem, traveler problem, network routing, and other optimization combination problems. Related scholars at home and abroad improve the ant colony algorithm; the most classical one is the maximum-minimum ant colony system (MMAS), which mainly improves three aspects, such as initializing the amount of information *τ*_*it*_(0)=*τ*_max_, to find the ant releasing pheromone of the shortest path after one cycle and limiting *τ*_*it*_(0) between *[Tmin, Tmax]*. The main parameters are chosen as follows: information heuristic factor *a*, expectation heuristic factor *β*, ant colony size *m*, and information volatility factor *p*.

(4) $$\begin{array}{c} \alpha \in \left[0,5\right],\\ \beta \in \left[0,5\right],\\ m\in \left[10,10000\right],\\ \rho \in \left[0.1,0.99\right]. \end{array}$$

*Calculation Method: Variable Initialization*. Determine the range of the study; *n* denotes the number of regions; that is, the range of the study is *n* regions. Create a matrix of weights for *n* regions, and the weights, namely, pheromones, are expressed in terms of EV traffic flow on each traffic path and specify the distance of each shortest path. Perform iterations. Specify the maximum number of iterations, and when the maximum number of iterations is reached, the iteration stops, and the best route and its distance are recorded. The probability of ants choosing a route is the probability that the charging station is set in a certain path, and the probability is calculated by the formula *b*_*i*_=(*τ*_*it*_/∑*τ*_*it*_) × *R*_*i*_. The preliminary station setting scheme is determined according to the probability size. According to the constraints in the model, if the conditions are met, the calculation continues to the next step, and if not, the probability is recalculated to determine the new station setting scheme. Select the path according to the objective function. Bring the number of site settings that meet the conditions into the model objective function, take the maximum value, and record the best path and update the pheromone. Continue the drop generation until the number of drop generations reaches the maximum value and stop. Get the best station setting value.

### 3.2. Landscape Evaluation of Public Charging Facilities

To evaluate the landscape design effect with high precision, an optimal landscape evaluation index system must be established. In this paper, a landscape evaluation index system is established based on the principles of representativeness, measurability, comparability, validity, and scientific, as shown in Table 1.

The quantitative operation of the landscape design effect is carried out in the form of a 100-point system, and they are described specifically as shown in Table 2.

We use the hierarchical analysis method to determine the weights of landscape design assessment indexes, and the specific process is as follows: (1) The landscape design effect assessment indexes are quantified and the judgment matrix of landscape design effect assessment indexes is established, as shown in the following equation:

(5) $$\begin{array}{c} \bar{A}=\left[\begin{array}{cccc} a_{1,1} & a_{1,2} & \cdots & a_{1,m}\\ a_{2,1} & a_{2,2} & \cdots & a_{2,m}\\ \cdots & \cdots & \cdots & \cdots \\ a_{m,1} & a_{m,2} & \cdots & a_{m,m} \end{array}\right], \end{array}$$

where *a*_*i, j*_ is the relative weight of indicator *i* relative to *j*. (2) Calculate the product of the elements of each row of equation (5); that is,

(6) $$\begin{array}{c} M_{i}=\prod_{j=1}^{n}a_{ij}. \end{array}$$

(3) Calculate the *n*th root of *M*_*i*_:

(7) $$\begin{array}{c} {\bar{w}}_{i}=\sqrt[{n}]{M_{i}}. \end{array}$$

(4) Normalize *w*_*i*_ using the following equation to obtain the weight vector as $\bar{w}={\left[w_{1},w_{2},\ldots ,w_{n}\right]}^{T}$.

(8) $$\begin{array}{c} w_{i}=\frac{{\bar{w}}_{i}}{\sum_{i=1}^{n}{\bar{w}}_{i}}. \end{array}$$

### 3.3. Design Algorithm of Public Charging Facilities in Ecological Landscape

The number of input, implicit, and output nodes of the BP neural network are *N, L*, and *M*, respectively. The structure of the neural network is shown in Figure 4. The input vector is *X*=[*x*_0_, *x*_1_,…, *x*_*N*−1_]; the weights between the implicit layer point *j* and the input layer point *i* and the output layer node *k* are *V*_ij_ and *W*_ik_, respectively, and the thresholds of the output and implicit layers are *ϕ*_*j*_ and *θ*_*k*_. The outputs of the nodes in the implicit layer and the output layer are computed as

(9) $$\begin{array}{c} h_{j}=f\left(\beta_{j}\right)=f\left(\sum_{i=0}^{N-1}V_{ij}x_{i}-\phi_{j}\right),\\ y_{k}=f\left(a_{k}\right)=f\left(\sum_{i=0}^{L-1}W_{ij}h_{i}-\theta_{k}\right). \end{array}$$

Calculate the deviation of *y*_*k*_ from the target output; that is,

(10) $$\begin{array}{c} \delta_{k}=\left(d_{k}-y_{k}\right)y_{k}\left(1-y_{k}\right),\\ \delta_{k}^{*}=h_{j}\left(1-h_{j}\right)\sum_{k=0}^{M-1}\delta_{k}W_{jk}. \end{array}$$

The weight adjustment size is calculated as

(11) $$\begin{array}{c} \Delta W_{jk}\left(n\right)=\eta \delta_{k}h_{j},\\ \Delta V_{ij}\left(n\right)=\eta \delta_{j}^{*}x_{i}. \end{array}$$

The adjustment of weights is given as

(12) $$\begin{array}{c} W_{jk}\left(n+1\right)=W_{jk}\left(n\right)+\Delta W_{jk}\left(n\right)+\mu \Delta W_{jk}\left(n-1\right)V_{ij}\left(n+1\right)=V_{ij}\left(n\right)+\Delta V_{ij}\left(n\right)+\mu \Delta V_{ij}\left(n-1\right). \end{array}$$

*Landscape Design and Evaluation Process*. (1) Establish the index system for landscape design evaluation. (2) Use hierarchical analysis to determine the weights of the indicators for landscape design assessment. (3) Collect sample data for landscape design assessment and use experts to score the effect of landscape design assessment, and form a sample set with its landscape design assessment indexes. (4) Adopt the number of landscape design assessment indicators to determine the number of input nodes of BP neural network, landscape design assessment effect as the output of BP neural network and determine the number of implied nodes of BP neural network according to certain formula so as to establish the topology of BP neural network. (5) Initialize the relevant parameters of the BP neural network. (6) Adopt the BP neural network to learn the training samples for landscape design evaluation and determine the optimal parameters with the landscape design evaluation accuracy as the training target. (7) Establish a landscape design assessment model according to the optimal parameters and test the model performance using the landscape design assessment test sample. The specific process of landscape design assessment by hierarchical analysis method and neural network is shown in Figure 5. The main steps include establishing the evaluation system and data collection, determining the BP neural network structure, and training the network. Finally, the performance of the model is tested using a landscape design evaluation test sample.

## 4. Experiments and Results

### 4.1. Experimental Setup

To test the performance of the hierarchical analysis method and neural network for the design and evaluation of ecological landscape public charging facilities, specific experiments were used to test their performance, and their measurement environment is shown in Table 3. To make the landscape design evaluation results of hierarchical analysis method and neural network comparable, the landscape design evaluation of hierarchical analysis method and landscape design evaluation method of BP neural network are selected for comparison test, and the evaluation accuracy and evaluation time are selected as performance evaluation indexes. The method proposed in this paper performs 30 epochs on the training dataset. The specific training method is as follows: the initial vector is set to 0.0001; the Adam optimizer is used; and the batch size is set to 8 (the batch size is the size of a training sample selected and the limitation of the device GPU to choose the best optimization and speed according to the model). The training process performance improvement and loss convergence diagram is shown in Figures 6 and 7. Analysis by Figures 6 and7 shows that a total of 30 epochs are trained, and the overall performance of the training process improves smoothly, and the model performance improves faster after 14 epochs, and the final accuracy converges to 99%.

### 4.2. Test Objects

For the effect of 50 ecological landscape public charging facility design solutions, multiple experts were used, and multiple peers scored according to the values of landscape design indicators as well as their own experience and knowledge, and the results of each landscape design scoring were counted, as shown in Figure 8.

From Figure 8, it can be found that the scoring results of different ecological landscape public charging facility design effects are different, indicating that the ecological landscape public charging facility design effects are characterized by certain randomness and nonlinear changes.

### 4.3. Comparison of Evaluation Accuracy of Indicator Layer

Ten ecologies landscape public charging facility design solutions were randomly selected as test samples and others as training samples, and five simulation tests were conducted for each method to reflect the fairness of the experimental results, and the accuracy of landscape design effect assessment is shown in Figure 9.

Comparing the accuracy of ecological landscape public charging facility design with Figure 9, we know that the average accuracy of ecological landscape public charging facility design of this paper is 91.52%, that of hierarchical analysis is 84.20%, and that of BP neural network is 86.3%. Compared with the comparative methods, the error of the ecological landscape public charging facility design effect assessment of this paper decreases significantly, which is mainly because the method of this paper integrates the advantages of hierarchical analysis and neural network, solves the defects of the current landscape design effect assessment with large errors, and verifies the superiority of the landscape design effect assessment method of this paper.

### 4.4. Ecological Landscape Charging Efficiency

According to the queuing theory model and the determined parameters, the charging stations and the installed charging piles are coded to generate the initial population, and then the dominant individuals are identified and entered the next generation of genetic operation based on the requirement of the least queuing time of the objective function. After a series of iterations, the final solution for selecting the location of charging stations and allocating the number of charging piles to make the objective function optimal is generated. According to the problem of charging station service efficiency, the number of populations, the length of individuals, the maximum number of iterations, the crossover rate, and the variation rate are 10, 9, 20, 0.8, and 0.01, respectively, when the number of charging stations is 120, 150, and 180, and the software is used for the programming operation of the ant colony algorithm. The basic process mainly includes the following steps: coding, creating the initial population, guiding the direction according to the fitness value after iteration, selection, crossover, variation, substitution to calculate the objective function value, and outputting the optimal solution. *Result Analysis*. When the number of charging posts is set to 120, the objective function value reaches the optimum at the 14th iteration and the least time is used (as shown in Figure 10). From the whole process of the change of the objective function value and the number of genetic iterations, the construction of the model and the selection of parameters are more scientific, and the objective value shows a continuous decline. Through simulation, it can be concluded that when 9 cells such as h1, h2, h3, h4, h5, h6, h7, h8, and h9 are selected to build stations, and the numbers of their charging posts are assigned as 16, 22, 15, 13, 5, 14, 11, 9, and 15, respectively; the total time consumption that can be achieved is 226.83, as shown in Table 4.

From the above table, the selection of 9 traffic districts for setting charging stations makes the ecologies landscape public charging facilities more widely radiated to all areas. The effect of neural network on the ecological landscape of charging facilities is shown in Figure 11. The decentralized layout of ecological landscape public charging facilities shortens the time consumed by users in the whole process of charging, makes it possible to get charging services nearby, saves the time of detouring and queuing, optimizes the network system, and maximizes the utilization rate of charging facilities and user satisfaction.

## 5. Conclusion

Landscape design is an important part of public charging facilities, and the functionality of the facilities nowadays is much more than the landscape. The application of landscape design in public charging facilities has not been explored to coordinate the environment, the value carried by the landscape itself, and the application of landscape design in public charging facilities. The combination of landscape design and base station is the protection and improvement of the living environment so that the ecological concept is used in the space: “The intelligent person hears in silence, and the wise person sees in the unformed.” The sustainable development of the charging station lies in the coprogression of the thinking of the times and environmental protection consciousness, reflecting the spirit of different places and social connotation in the ecological consciousness. In the present era of pursuing low carbon and environmental protection, public charging facilities in cities will certainly become an indispensable part. In addition to the main charging function, the principles and concepts of its landscape design have positive marketing to the urban living environment and can play the role of embellishment. The human-oriented design concept should be applied to give it better convenience and functionality, better meet the public demand in the information age, realize greater value, create a more harmonious and beautiful urban environment, add fun, and facilitate people's daily life.

In response to the defects in the current evaluation process of ecological landscape public charging facility design, based on the theory of combinatorial optimization and using the respective advantages of hierarchical analysis and neural network, we propose a landscape design effect evaluation method of hierarchical analysis and neural network, using hierarchical analysis to establish a scientific and objective evaluation index system of ecological landscape public charging facility design and using the nonlinear fitting ability of neural network. Tracking the changing characteristics of landscape design, they overcome the defects of single hierarchical analysis method and neural network. The main steps of the proposed method are as follows: (1) establish the evaluation system and data collection; (2) determine the BP neural network structure; (3) initialize the neural network and train the network; and (4) build the landscape design evaluation model according to the optimal parameters and test the performance of the model using the landscape design evaluation test samples. The final test results show that this paper's method is a high-precision and fast landscape design effect assessment method, and the assessment results can provide valuable reference opinions for the design staff of ecological landscape public charging facilities, which has a very wide application prospect. In the future, we plan to conduct research on public charging facilities for electric vehicles based on knowledge mapping and recurrent neural networks that integrate landscape design and environmental protection.

## Figures and Tables

**Figure 1:** Diagram of the new demand analysis path for standardization of charging facilities in ecological landscapes.

**Figure 2:** The basic framework of habitat standardization system for electric vehicle charging facilities.

**Figure 3:** Overall model structure.

**Figure 4:** Neural network structure.

**Figure 5:** Landscape design evaluation process with hierarchical analysis and neural network.

**Figure 6:** Training process performance improvement diagram.

**Figure 7:** Training process loss convergence diagram.

**Figure 8:** Scoring value of landscape design effect.

**Figure 9:** Comparison of the accuracy of landscape design effect assessment by different methods.

**Figure 10:** Charging pile output results graph.

**Figure 11:** The effect of neural networks for ecological landscaping of charging facilities.

**Table 1:** Landscape design effect comprehensive assessment index system.

Target layer	Level 1 indicators	Level 1 indicators
Comprehensive assessment of landscape design effects	Scientific Artistic Protective	Overall conformity
		Functionality
		System integrity
	Economical Level 1 indicators Scientific	Natural aesthetics
		Space creation
		Vernacular culture
	Artistic Protective	Landscape pattern protection
		Vernacular culture preservation
		Conscious space preservation
	Level 1 indicators	Project cost
		Maintenance costs
		Landscape economic vitality

**Table 2:** Scoring criteria for comprehensive assessment results of landscape design effects.

Landscape design effect assessment grade	Score
Excellent medium	90–100
Qualified	80–90
Unqualified	70–80
Landscape design effect assessment grade	60–70
Excellent medium	60

**Table 3:** Test environment setup.

Parameter	Parameter values
CPU	AMD 3.0 GHz
RAM	16 GB
Hard disk	1000 GB SDD
Network card	1000M
Operating system	Win 10
Programming tool	VC6.0++

**Table 4:** Optimization results of charging facility site selection.

Charging station setup	Charging pile setup	Demand share (%)	Queuing time (h)	Detour time (h)	Total time consumption (h)
h1	(pcs)	13	50.61	176.22	226.83
h2	16	18			
h3	22	12			
h4	15	11			
h5	13	4			
h6	5	12			
h7	14	9			
h8	11	7			
h9	9	12			

## Data Availability

Data sharing is not applicable to this article as no new data were created or analyzed in this study.
